RETRACTED

# Detection and Application of Wearable Devices Based on Internet of Things in Human Physical Health

**DOI:** 10.1155/2022/5678736

**Published:** 2022-06-21

**Authors:** Jingjing Lou, Fan Yang, Changsheng Lv

**Affiliations:** ^1^Guangzhou Institute of Sports Science, Guangzhou 510620, Guangdong, China; ^2^Guangzhou Tianhe Sports Centre, Guangzhou 510620, Guangdong, China; ^3^Guangzhou Sports University, Guangzhou 510620, Guangdong, China

## Abstract

In order to improve the detection function of wearable intelligent devices in the Internet of things and facilitate people to control a variety of information such as heart rate, exercise state, blood oxygen saturation, and so on, the scientific detection of human physical health based on wearable devices based on Internet of things technology is proposed. Through the combination of software- and hardware-related functional modules, the real-time detection of human physical health information can be effectively realized. Firstly, the detection principle of optical capacitance product pulse wave signal and the waveform characteristics of pulse wave are introduced, and then the application scenarios and advantages of wearable devices are further introduced; then, the convolutional neural network for pulse wave signal denoising and the basic principle of self-encoder are introduced; finally, the regression prediction method and support vector machine method for pulse wave signal feature extraction are introduced in detail. The pulse wave based on optical capacitance product is removed to improve the waveform quality of pulse wave signal. Firstly, the system software development environment is briefly described. Then, the software design of watch terminal master device based on MSP432 and belt terminal slave device based on MSP430 are described in detail, and the detailed program implementation flow of each key technology in the system is given. In addition, the fall detection algorithm based on threshold discrimination is studied, and the program implementation of the algorithm is also described in detail. Finally, the system is tested. The results show that normal state mainly include normal walking, jogging, and fast sitting, and the accuracy rate is 97%, 95%, and 93%, respectively. For fall state, the experimenter needs to simulate various possible fall states, and the accuracy rate is 95%, 93%, and 95%, respectively, which verifies the detection accuracy of the algorithm. The system can automatically turn on the satellite positioning function when the user's physical sign parameters are abnormal or the user's current fall dangerous situation occurs, and send the current position information and alarm content information through the GSM module, so that the dangerous situation can be found and handled at the first time.

RETRACTED

## 1. Introduction

According to the relevant report data released by the World Health Organization in 2021, from 2010 to 2020, more than 60% of the causes of death in the global population were chronic diseases. Chronic diseases such as cardiovascular and cerebrovascular diseases, hypertension, diabetes, and respiratory diseases are often hard to detect. In addition, these diseases are often accompanied by sudden complications when they relapse, so the symptoms are hard to find in time. Taking respiratory diseases as an example, the detection of this disease requires real-time grasp of human heart rate changes, but the traditional treatment and prevention methods cannot detect human heart rate changes in real time, so long-term health level monitoring technology must be used [1]. With the continuous development of science and technology, especially the arrival of the era of intelligent terminals, there are more and more wearable devices, and the technology is becoming more and more perfect. Many wearable devices are widely used in the field of medical monitoring. With the help of wearable intelligent devices, various physiological characteristics of human body can be monitored in real time and unhealthy factors of human body can be found in time, as shown in Figure 1. It can be said that the emergence and technical improvement of wearable intelligent devices provide strong technical support for the realization of human long-term health monitoring. This paper focuses on the application of wearable devices in human physical health monitoring based on the Internet of things technology [2].

## 2. Literature Review

In recent years, wearable monitoring systems have been widely used in human daily life, such as entertainment, learning, health care, medical treatment, and so on. These devices can help people better understand and explain their living conditions. In the past few years, people have paid more and more attention to the mental health problems on university campuses. Some researchers have creatively studied some mental health problems by means of wearable sensors, mobile phones, and questionnaires. Han J. and others developed a machine learning algorithm based on wearable sensor data to distinguish college students' happiness and unhappiness. The algorithm can evaluate the relationship between different components of happiness, including happiness, health, energy, alertness, and stress [3]. However, there are still some problems in mental health monitoring, one of which is privacy protection. In addition, wearable monitoring system also has some challenges in long-term monitoring, real-time data calculation and analysis, portability, and effective evaluation.

RETRACTED

With the continuous development of big data technology, the auxiliary technology based on machine learning algorithm is widely used in a variety of diagnostic tasks. RR interval is one of the most popular time-domain features in the related diagnostic tasks of ECG signals. RR interval refers to the time interval between one heartbeat peak (r peak) and another. The change of heart rhythm can be effectively evaluated through RR interval. Lin T. et al. used RR interval as feature input into machine learning diagnosis model. By detecting the changes of blood vessel volume during heartbeat and respiratory activities, the pulse wave signal can indirectly reflect the functions of autonomic nervous system such as heart. The interval change between the two peaks of pulse wave has the same physiological significance as RR interval [4].

The health monitoring application based on wearable devices can be mainly divided into three aspects: autism monitoring for teenagers and children to help wearers find autism status earlier and create better treatment conditions; Medical and health monitoring for the elderly, through wearable devices to help the elderly remote medical monitoring, medical assistance, etc.; Surantha N. et al. focused on the behavior habit monitoring and psychological disorder monitoring of young people. The behavior habit monitoring mainly used wearable devices to monitor the exercise, social and other living habits of young people, and help the subjects solve problems such as alcoholism and obesity. The psychological disorder monitoring mainly included anxiety related to mental health, communication disorder caused by loneliness, early depression, and neurological symptoms [5].

At present, wearable consumer electronics products such as smart bracelets and smart watches in the consumer market can be described as a hundred flowers bloom, but most wearable devices usually only integrate behavioral motion sensors, which only realize a simple step counting function. Researchers mainly apply wearable devices to the field of personal health care and behavior recognition, such as health monitoring of the aging population. In terms of medical care, the pulse oximeter designed by Mekruksavanich S. et al. and the real-time gesture interaction system with multi-modal human-computer interaction function can not only monitor the health of the elderly but also monitor the physiological parameters such as ECG, heart rate, blood oxygen saturation, skin moisture, body fat content, and so on [6]. Karthick G. S. et al. have made substantial progress in remote monitoring. They designed and implemented a wearable real-time monitoring terminal for ambulatory ECG based on the Internet of things, connected it to the Internet through the gateway, and then sent the collected sensor data to the cloud server. This system can collect, analyze, and alarm ambulatory ECG signals in real-time [7]. Chen I. Z. et al. developed a wearable multi physiological parameter health monitoring system, and built a complete set of medical auxiliary monitoring system by using wearable clothes, reflective pulse sensor, and physiological signal acquisition module, which can be applied to the field of medical care [8]. In the field of behavior recognition, Sa Nn Ino G. et al. used chest sensors, wrist sensors, and ankle sensors to collect behavior data sets, and built a human daily behavior recognition model based on the integrated learning model algorithm [9]. Msr A. et al. have done a lot of research work in a research direction of human-computer interaction and pervasive computing (user activity recognition), and applied motion sensor recognition technology, sound sensor recognition technology, and other physiological index sensor recognition technology to daily activity recognition [10]. Kyriakopoulos G. et al. took the lead in applying wearable devices to the research field of College Students' mental health. They monitored 30 participants for two weeks, counted the students' sleep, diet, and stress levels through the Panas scale, collected the behavior data of the experimental subjects through Fitbit exercise bracelet, and finally found that eating habits may affect the students' stress, sleep, and exercise [11]. Xing F. et al. also conducted a 30-day research experiment on 66 participants using wearable sensors and smart phones to explore the correlation between academic performance (GPA), Pittsburgh sleep quality index (PSQI), perceived stress scale (PSS), and mental health comprehensive SF-12 score (MCS). These objective data were used for machine learning model training, and the classification accuracy was 67–92% [12]. Based on the current research, this paper proposes the scientific detection of human physical health based on wearable devices based on Internet of things technology. Through the combination of software- and hardware-related functional modules, it can effectively realize the real-time detection of human physical health information. Firstly, the heart rate acquisition module and fall detection module are experimentally verified, and the results are analyzed in detail. Finally, the commissioning test of the whole system is completed to verify the abnormal alarm mechanism of the system. In the research and design of the system, at present, the basic human body sign information data collection and fall detection are completed, and the positioning and alarm information are sent to achieve the expected goal of the subject.

RETRACTED

## 3. Overview of Relevant Technologies

### 3.1. Optical Capacitance Pulse Wave and Wearable Devices

The basic measurement principle of PPG technology comes from the refraction and reflection of light. According to the Lambert Beer law, when light shines on the target medium, it will absorb light to varying degrees due to different object materials and densities. When light irradiates the tested human body with a certain intensity and wavelength, a small area composed of bone, skin, venous blood, arterial blood, and other tissues can be regarded as a medium with fixed structural components. Therefore, the amount of light absorption and reflection is fixed. The amount of light absorption will change only when the blood volume in the blood vessel changes. Since the change of light absorption is directly proportional to the change of blood volume in the blood vessel, the pulse wave waveform can be detected by detecting the change of light absorption when it irradiates the target object through the photoelectric detector [13].

Pulse wave signal contains rich information of human physiological conditions, with representative wave characteristics. The appearance of a wave peak represents a process of cardiac contraction. During a contraction of the aorta, blood is injected into the heart [14]. One point represents the end of the cardiac ejection process, followed by the descending branch, that is, the process from the end of one cardiac ejection to the beginning of the next ejection. This period of time accounts for a long period of the whole pulse wave, because after the ejection process, the arterial blood is injected into the aorta in a tidal way, and the two points correspond to the regression process after the blood strikes the vascular wall, which is also called heavy wave front wave. Point 3 and point 4 represent the trough and peak of heavy wave, respectively. After the completion of ejection, the change of blood flow in blood vessels gradually slows down, so the peak value 4 is significantly less than point 1. This is because after the heart completes the ejection process, the aortic valve will close, and after the blood impacts the vascular membrane wall, it will have a reverse impact due to the impact on the vascular wall [15].

### 3.2. Convolutional Neural Network

The ANN of the foundation is mainly composed of input layer, middle layer, and output layer, and each layer is fully connected. A single neuron in the input layer represents the characteristics of an input data. The number of neural network units in the output layer is usually determined by the specific target task. If it is a classification task, the number of output layers corresponds to the number of classification labels. The hidden unit in the middle is determined according to the dimension of feature learning. After designing the model structure according to the task goal, the optimal solution of the target task can be found through the gradient descent algorithm. With the emergence of big data technology and massive data, scholars fully learn the potential characteristics of input signals by stacking multi-layer ANN. The multi-layer neural network structure can mine the relationship between input data and machine learning tasks by expanding the hidden layer of neural network, so as to fully learn the high-dimensional features of data. Compared with traditional neural networks, CNN uses convolution layer instead of full connection layer, which greatly reduces the number of parameters in the model network. Moreover, through the design of pooling layer and residual network, it can not only greatly reduce the amount of calculation in the process of model training but also increase the depth of the model according to the task objectives, which has good scalability [16].

RETRACTED

### 3.3. Self-Encoder

AE is an unsupervised learning algorithm mainly used for data dimensionality reduction or feature compression, which can reproduce the dimensions and features of input data at the output layer. In order to realize the reproduction of input data, it is necessary to capture the representative characteristics of input data in the middle layer and identify the main components of input data. Therefore, the number of neurons in the middle layer is usually smaller than that in the input and output layers.

The self-encoder is mainly composed of encoder and decoder. The input data *x* has the same dimension as the output data *y*. The encoder first compresses the input data into hidden layer features, and then reconstructs the output through the features. In the encoder part, the function *f* (*x*) maps the input data *X* to the hidden layer feature representation *h*:

(1) $$\begin{array}{c} h=f\left(x\right)=\omega_{f}\cdot x+b_{f}, \end{array}$$

where *ω*_*j*_ and *b*_*j*_ are the neural network parameters to be learned. Then, let *y* represent the reconstructed output, and g (*h*) represent the function corresponding to the decoder. Its function is to reconstruct the hidden layer feature *h* into the output *y*. The decoder function can be defined as:

(2) $$\begin{array}{c} y=g\left(h\right)=\omega_{g}\cdot h+b_{g}. \end{array}$$

We can use the mean square error as the loss function of the self encoder:

(3) $$\begin{array}{c} L\left(\omega ,b;x\right)=\frac{1}{n}\sum_{i=1}^{n}{\left\|g\left(f\left(x_{i}\right)\right)-x_{i}\right\|}^{2}. \end{array}$$

The training process of the self-encoder is to continuously adjust the network parameters to minimize the reconstruction error between *X* and *y*. After two model processing steps of encoding and decoding, the self encoder first compresses *x* into H, and then reconstructs it into *y*. Because the data dimension of the middle hidden layer is usually smaller than the input data dimension, the feature expression vector *h* of the hidden layer realizes the coding volume reduction and feature compression of the input features [17, 18].

RETRACTED

### 3.4. Regression Prediction Method

Linear regression refers to the fact that the regression model is composed of linear variables. It is the preferred target model for a prediction task. In the prediction task, the dependent variable is usually required to be continuous, and the independent variable can be continuous or discrete. Finally, the relationship between the independent variable and the dependent variable is established through function fitting. Regression method can also be used in binary classification tasks, in which the output value of binary classification is only yes or no, or 0 and 1. Its essence is to use threshold method to segment the output results on the basis of linear regression.

There are many fitting methods for multiple input features. As the basic model of statistics, multi dependent variable linear regression method is widely used in various analysis tasks. Assuming that *x* = [*x*1, *x*2, ..., *xn*] with input feature dimension *n* has a certain linear relationship with output *Y*, then:

(4) $$\begin{array}{c} Y^{\prime }=\beta_{0}+\beta_{1}x_{1}+\beta_{2}x_{2}+\cdots +\beta_{n}x_{n}. \end{array}$$

As shown in formulas (5) and (6), we usually represent the loss function by the error between the actual value of the sample and the output value of the model:

(5) $$\begin{array}{c} L\left(\beta \right)=\frac{1}{2}{\left[Y^{\prime }-Y\right]}^{2}=\frac{1}{2}{\left[\beta_{0}+\beta_{1}X_{1}+\beta_{2}X_{2}+\cdots +\beta_{n}X_{n}-Y\right]}^{2}, \end{array}$$

(6) $$\begin{array}{c} L\left(\beta \right)=\frac{1}{2}{\left[Y^{\prime }-Y\right]}^{2}=\frac{1}{2}{\left[\beta^{T}X-Y\right]}^{2}. \end{array}$$

After determining the form of loss function, the regression coefficient is usually solved by minimizing the loss function. There are two methods to minimize the loss function: least square method and gradient descent method. The essence of the least square method is a process of finding the extreme value, which can be solved by calculating the partial derivative of the regression coefficient. The gradient descent method is also to solve the gradient descent direction of the function by calculating the partial derivative, and continuously updating the target value according to the iterative step size until the algorithm reaches the acceptable error range. The formula for partial derivative of regression coefficient is as follows:

(7) $$\begin{array}{c} \nabla L\left(\beta \right)=\nabla \beta \frac{1}{2}\left[{\left(\beta^{T}X-Y\right)}^{2}\right]=\nabla \beta \frac{1}{2}\left[{\left(X\beta -Y\right)}^{T}\left(X\beta -Y\right)\right],\\ \nabla L\left(\beta \right)=\nabla \beta \frac{1}{2}\left[{\left(\beta^{T}X-Y\right)}^{2}\right]=X^{T}X\beta -X^{T}Y, \end{array}$$

where, let the partial derivative ∇*L*(*β*)=0 to calculate the value of the regression coefficient as follows:

(8) $$\begin{array}{c} \beta ={\left(X^{T}X\right)}^{-1}X^{T}Y. \end{array}$$

The least square method requires that the optimal estimation of the model can be obtained only when the assumptions are strictly met, but there are often problems in the actual problem scenario [19, 20]. For example, variables are seriously disturbed by anomalies, variables are missing, and variables come from different probability distributions. Therefore, it is necessary to design a more robust regression scheme in combination with relevant algorithms.

RETRACTED

### 3.5. Support Vector Machine

Support vector machine (SVM) is a kind of machine learning model based on statistical theory. Its advantage lies in small sample learning and high-dimensional feature learning of input data. The design idea of SVM is to map the input data to a higher dimensional space by selecting an appropriate kernel function, and find a hyperplane to separate multiple types of data as much as possible. For the classification problem, the principle of SVM is to maximize the classification interval as much as possible on the premise of ensuring the classification accuracy. Take the simplest binary classification as an example. For the input variable *x*, we use *y* to represent its input result:

(9) $$\begin{array}{c} y=\omega \cdot x+b. \end{array}$$

Figure 2 shows such a linear separable problem in two-dimensional space. Blue dots and red dots represent positive samples and negative samples, respectively. The goal of SVM is to find a red classification line as shown in the figure to perfectly separate the two types of samples. Among them, *y* = −1 and *y* = 1 represent the two positive and negative samples closest to the classification line, also known as support vector. The selection of support vector is very important for the classification task. The auxiliary solution of classification line can be carried out through support vector [21]. When the two-dimensional space corresponding to the simple binary classification problem is extended to the high-dimensional space, it is not the category that the classification line can solve. At this time, the problem is to find a target hyperplane and separate the classification samples in the form of maximum spacing. The target formula is as follows:


(10) $$\begin{array}{c} \min\frac{1}{2}{\left|\omega |\right|}^{2},\\ \text{s.t.}\left\{\begin{array}{c} y_{i}\left(\omega \cdot x_{i}+b\right)-1\geq 0,\\ i=1,2,\ldots ,l. \end{array}\right. \end{array}$$

Since most samples in reality are linearly inseparable, in order to solve the problem of linearly inseparable in the actual scene and increase the fault tolerance rate of samples, a new relaxation variable is added to the model, and then the target formula is rewritten as:

(11) $$\begin{array}{c} \min\frac{1}{2}{\left|\omega |\right|}^{2}+C\sum_{i=1}^{i}\xi_{i},\\ \text{s.t.}\left\{\begin{array}{c} y_{i}\left(\omega \cdot x_{i}+b\right)\geq 1-\xi_{i},\;\left(i=1,2,\ldots ,l\right),\\ \xi_{i}\geq 0,\;\left(i=1,2,\ldots ,l\right). \end{array}\right. \end{array}$$

For the solution of the above problems, we usually convert the above formula into a dual problem with the help of Lagrange algorithm. The specific process is to first convert the above formula into Lagrange function:

(12) $$\begin{array}{c} L\left(\omega ,b,\alpha ,\beta \right)=\frac{{\left|\omega |\right|}^{2}}{2}+C\sum_{i=1}^{i}\xi_{i}-\sum_{i=1}^{i}\beta_{i}\xi_{i}-\sum_{i=1}^{i}\alpha_{i}\left[y_{i}\left(\omega \cdot x_{i}+b\right)-1+\xi_{i}\right]. \end{array}$$

Next, the model parameters can be solved by calculating the partial derivative of each parameter. In the SVM classification task, the selection of kernel function is also a very important content. The kernel function determines the way to map the input data to the high-dimensional space and convert the nonlinear problem into a linear problem to solve it. Therefore, selecting an appropriate kernel function is conducive to further improve the accuracy and stability of the classification task.

RETRACTED

## 4. System Software Design and Implementation

### 4.1. Noise Reduction Based on Optical Capacitance Product Pulse Wave

Due to the complexity and diversity of practical application scenarios, the optical capacitance product pulse wave signals collected by wearable devices are usually disturbed by the surrounding environment, light, motion artifacts, and other noise [22]. Before further feature extraction and health monitoring tasks, the waveform quality of pulse wave signal should be improved by removing noise components. Traditional signal denoising schemes include wavelet transform, singular value decomposition, and so on. Single method or combination can effectively remove the interference of some noise. When there is no frequency band overlap between the noise interference and the characteristic signal, the traditional signal processing method performs better, mainly filtering the noise interference outside the target frequency range through spectrum analysis and signal filtering. However, when there is co frequency interference, the traditional method is difficult to play an effective role. For example, in the actual scene, the interference of motion artifacts is very difficult to filter out, and the frequency range of motion artifacts is easy to coincide with the frequency range corresponding to respiratory rate and heart rate [23]. When the noise has a great impact on the waveform quality of pulse wave signal, it will greatly affect the accuracy of subsequent feature extraction, which is not conducive for further physiological feature parameter extraction and health level anomaly detection.

#### 4.1.1. Noise Reduction Self-Encoder Network

The noise reduction self coding model is mainly composed of encoder and decoder. The input and output data have the same dimension. The training process of self-encoder takes the real signal as the input directly. Therefore, when the input contains noise, it will produce the possibility of over fitting, so as to reduce the learning ability of the model for the input data. In complex cases, considering the difference of each sample and the influence of noise, similar samples will not show strictly the same characteristics. This requires that the neural network has robustness and strong generalization ability. DAE is to artificially introduce noise into the input data to solve the above problems. Specifically, by adding a certain proportion of noise to the original input data, the obtained noisy data set is used as the input of the encoder, and the data are reconstructed at the output of the decoder [24]. By introducing noise, the model has certain anti noise processing ability for noisy signals. In the DAE model, the initial input *x* is destroyed into *x* by introducing random noise. The loss function shown in formula (13) can be rewritten as:

(13) $$\begin{array}{c} L\left(\omega ,b;\tilde{x},x\right)=\frac{1}{n}\sum_{i=1}^{n}{\left\|g\left(f\left({\tilde{x}}_{i}\right)\right)-x_{i}\right\|}^{2}. \end{array}$$

In the DAE model, the hidden layer unit has smaller dimensions than the input-output layer. The design can well extract the hidden feature *h* of input *x*, and then map it to the corresponding reconstructed output *y*. Since the popularity of deep neural network, the stacked structural design of DAE model has appeared. Stacked DAE is composed of multi-layer neural network structure, which can extract deep-seated high-dimensional features. The output of each layer in the hidden layer is used as the input of the next layer. This model obtained by stacking hidden layers is called stacked DAE. The hidden layers of stacked DAE are usually fully connected, but CNN can be used as the basic hidden layer network structure for the data with periodic regular changes taking pulse wave signal as an example. CNN is first used in image and natural language processing, and then attracted much attention because of its superior performance in extracting local features. CNN is also suitable for feature learning of time-series periodic signals. There are some differences between the noise reduction self-encoder network based on CNN and the traditional stacked DAE. The former uses convolution layer and pooling layer instead of full connection layer in the encoder. Compared with other models, the model based on convolution neural network shares fewer parameters, which can better extract the characteristics of input data and reduce the amount of calculation in the training process. To sum up, the noise reduction self-encoder is a special self-encoder model by introducing random noise into the input layer [25]. The model can not only fully learn the potential characteristics of the signal but also better learn the characteristics of the target signal and noise interference, and effectively recover the original signal characteristics from the damaged input signal. The introduction of noise can help to improve the robustness of the model. In the presence of noise interference, it can still denoise the signal according to the learned signal characteristics and noise characteristics. It is expected to realize the denoising and effective information reconstruction of pulse signal in complex environment.

RETRACTED

Select 80% of the pulse signal records as the data set used in the training process and the other 20% as the data used in the prediction process, so as to ensure that there is no cross between the training set and the prediction set. For the unlabeled nonnoise control data and labeled noisy input data used in training, we will further randomly divide the training set and test set, in which the test set and training set do not intersect in each round of training, but the test set may contain historical pulse wave WaveForms of the training set, while the data in the prediction set come from different pulse wave records. In the process of model training, we use the cross validation method as the scheme to evaluate the denoising performance of the model. Specifically, all the training data sets are divided into 10, of which 9 are used as the training set for model optimization and the other as the test set for model effect verification. The test set and training set are randomly divided after data confusion.

Table 1, Figures 3 and 4, respectively, show the results of signal denoising for randomly superimposed baseline drift, EMG interference, and electrode interference noise used to simulate motion artifacts. From the model denoising results, we can see that because the test set contains the historical waveform in the model training process, and the prediction set has no intersection with the model training data set, the denoising effect of the model in the test set is generally better than that of the prediction set. Although the prediction set does not intersect with the training, it has similar characteristics in waveform. Therefore, for the new signal characteristics in the prediction set, SCDAE model also shows better signal denoising ability.

#### 4.1.2. Comparison of Denoising Performance with Traditional Methods

In order to verify the effectiveness of the deep noise reduction network proposed in this paper, this paper selects the form of comparison with the traditional denoising methods to show the performance of the model. The control group of the experiment is divided into traditional method and neural network model. Among them, there are two groups of traditional methods, SVD and WT, which denoise the pulse wave signal through the combination of traditional methods. The neural network model control group is a five layer network structure DDAE with full connection mode, which is used to compare the effectiveness of the model and optimization method based on convolutional neural network. In the control group of traditional methods, in order to improve the calculation efficiency in the filtering process and retain the effective information in the pulse wave signal as much as possible, firstly, the high pass filter is used to remove the extremely low-frequency noise. Specifically, the Chebyshev II filter is used to remove the extremely low-frequency noise interference below 0.1 Hz. Wt group used discrete wavelet transform to decompose the pulse wave signal in seven layers, and selected A7, D5, D6, and other components for signal reconstruction. SVD group uses the combination of discrete wavelet transform and singular value decomposition to denoise the signal with finer granularity. The data set used in the experimental group of traditional methods is consistent with the test set data mentioned above in quantity, and 20% of the original data are randomly selected for signal denoising and performance evaluation [26].

RETRACTED

Figures 5 and 6, respectively, show the experimental results of SNR and *R* coefficient after signal denoising. In order to facilitate and intuitively display, the experimental results of SCDAE model and three control groups are compared in the form of histogram. In the experimental design, the two groups of deep learning evaluate the denoising performance of pulse wave signal on the test set and prediction set, respectively. Taking the SCDAE model designed in this paper as an example, SCDAE_t represents the test set and SCDAE_p represents the prediction set. From the figure, we can see that for the two traditional methods, the overall performance of the SVD group is better than that of the WT group, and SVD has more fine-grained decomposition in signal denoising. However, both SVD and WT perform poorly in removing motion artifact noise. This is because there is a large amount of overlap between motion artifact and pulse wave signal spectrum, which will simulate P wave or destroy the waveform characteristics of heavy pulse wave to a certain extent, resulting in artifacts.

At the same time, it enhances the scalability of the model and shows the best performance on the same data set. In general, when there are many kinds of complex noises in the environment, the deep noise reduction network method based on convolutional neural network shows good signal denoising and reconstruction performance, and is suitable for tasks requiring high waveform quality. In the context of big data medical treatment, a monitoring scheme for personal health level is designed. Combined with the characteristics of similar characteristics between personal historical data samples, pulse wave signal denoising and further feature extraction are carried out.

### 4.2. Software Platform Development

In the engineering practice of debugging and downloading microcontroller MCU software, the most used development tools mainly include IAREmbeddedWorkbench (IAREW) of IARSystems company and CCS6.1 of TI company. In this software development process, IAREmbeddedworkbench is the main development environment and CCS6.1 is the auxiliary development software; the emulator selected for MSP432 software debugging is XDS110-ET, and the emulator selected for MSP430 software debugging is MSP-FET430UIF.

The development process of the software part mainly includes the overall design planning of the software, the compilation of source code, and online simulation debugging and system debugging. After continuous modification and debugging, the expected goal is achieved. The specific software development process is shown in Figure 7.

RETRACTED

### 4.3. Software Design of Main Equipment

The subroutine design of MSP432 mainly includes the main equipment system initialization configuration program design, A/D conversion subroutine design, Bluetooth communication subroutine design, IIC communication subroutine design, and corresponding IO port configuration. The software design block diagram of wristband terminal node based on MSP432 is shown in Figure 8.

The wristband terminal based on MSP432 exists as the master device in the whole system. After the master device is powered on and works normally, it will read whether the user has enabled the option of establishing Bluetooth connection. If the option of establishing Bluetooth connection is enabled, search the Bluetooth signal of the slave device and pair the connection, and read the relevant human posture information uploaded from the device. At the same time, MSP432 reads the relevant sign information collected by the physiological sensor to analyze and judge whether the current user is abnormal. In case of abnormality, the system delays for 30 s, and the user can judge whether it is a misjudgment. If it is a misjudgment, the alarm information can be manually closed through the equipment button; if it is determined that the user is currently abnormal, the system will automatically start the positioning module to determine the current location information, and send the current abnormal information and location information to the designated person through the GSM module; in this process, if the user does not turn on the option of establishing Bluetooth connection, the main device will turn off BLE4.0 module to reduce the power consumption of the device. MSP432 will only analyze the relevant sign information collected by the physiological sensor, and send the relevant information to the designated person at the first time when it is confirmed that the user's sign parameters are abnormal.

IIC communication mode is adopted for OLED screen module, heart rate acquisition module, and micro power consumption meter in the main equipment system. IIC bus is a two wire serial communication bus protocol launched by Philips in the early 1980s. It has the characteristics of simple interface and high communication rate, so it is widely used. IIC bus consists of two communication lines: serial data line SDA and serial clock line SCL. IIC bus is a half duplex communication bus, so the two-way communication of data can be realized between MCU and the device controlled by IIC. According to different data transmission rates, IIC bus can be divided into three communication modes with different rates, namely, standard mode (100 kbit/s), fast mode (400 kbit/s), and high-speed mode (3.4 mbit/s). In the slave communication mode, the main controller MCU and multiple IIC bus devices are allowed to be mounted on the same IIC bus to realize data exchange. In the specific communication process, different communication objects are identified by the device address.

RETRACTED

In the process of IIC communication, the host initializes the IIC bus and generates clock SCL signal, while the slave is an addressed unit in the bus, which is mainly responsible for data acquisition and waiting for the request instruction sent by the host. In the whole IIC communication process, the start and stop of data transmission are controlled by the host. When the IIC bus is idle, the data line (SDA) and clock line (SCL) are set to high level; when the data transmission is started, the clock line is first pulled high, and the data line generates a negative jump signal from high to low, and starts to send data; the host will generate a reply ACK signal after receiving the data sent by the slave. If the reply is not generated, continue to wait for a new start signal; when the data transmission is completed, the clock line will be pulled up again, and the data line will generate a jump end signal from low to high. At this time, the IIC bus is idle again. In the process of IIC bus data transmission, when the clock line is at high level, the data transmitted on the data line SDA must remain relatively stable. Only when the clock signal is at a low level, the level state on the data bus can be changed.

The wireless data communication between the master and slave devices of the system is carried out through Bluetooth 4.0. The Bluetooth transmission must go through the following four steps: searching the device, establishing connection, pairing, and binding. The specific Bluetooth transmission process is as follows:

1. The slave device first sends a broadcast signal (including equipment address, equipment name, and other relevant information), and the host device immediately sends a scanning request after receiving the broadcast signal; when the slave device receives the scanning request and correctly returns the response signal, the step of searching the device is completed correctly.
2. After completing the device search, it is necessary to establish a Bluetooth transmission connection line. The host device will send a connection establishment request, and the slave device will receive the connection establishment request and correctly return the establishment response signal, that is, complete the steps of establishing the connection.
3. In order to ensure the security of data in the transmission process, authentication is required first when some important data exchange is carried out. The specific verification process is as follows: When one party (either the host device or the slave device) accesses the other party's important data, it must first send the correct authentication password to the other party, and then access the other party's important data after verification. This verification process is called pairing.
4. The process of authentication each time is more troublesome. BLE4.0 protocol stack can save the authentication password between the master and slave devices, so that they can connect quickly the next time without re-authentication. This process is called binding.

RETRACTED

UART serial communication is used for data transmission between Bluetooth BLE4.0 module, GSM module, Beidou positioning module, and MSP432 in the main equipment system. UART is a full duplex universal asynchronous serial communication data bus, which can realize two-way transmission and reception of data. UART communication process is to send or receive the data to be sent or received by byte shift. The sending process of data is to first turn on the byte sending function to send the data in the byte frame from the low start bit, with 5–8 data bits in the middle. At the end of the byte frame, one available parity bit and one or more high stop bits are provided. The sending process of bytes is controlled by the sending end control register; the data receiving process is that when there is no data update in the byte receiving shift register, the bus controller will monitor the state of RXD data line by means of timing interrupt. When it is detected that the RXD bus level is 1, 0, and 0 for three consecutive times, the data transmission start bit, the shift register at the receiving end is ready to receive the data, the byte frame receiving process is controlled by the control register at the receiving end, and the byte receiving process data are still received in serial mode. During the initialization of UART serial port program, the data format of UART serial port communication is specified. Each data frame is 10 bits (1 start bit, 8 data bits, no parity bit, 1 end bit), and the transmission baud rate is set to 9600 characters/*s*. The core function of the system is to send relevant alarm information to the designated personnel and provide the current location of the user in case of abnormal dangerous situation. After the system is powered on, the master and slave devices are initialized, and the relevant peripheral function modules are also initialized. When the user's physical parameters are abnormal or the user is in danger of falling, the main equipment itself will generate an audible alarm and delay for a period of time to remind passers-by and the user. If the user does have a dangerous situation, the system will open the positioning module to determine the current position and send relevant alarm information through GSM module; if the current alarm generated by the equipment is a false alarm, the user can manually choose to turn off the alarm sound and stop the equipment from sending relevant alarm information.

RETRACTED

### 4.4. Fall Detection Algorithm and Program Implementation

Firstly, the human posture coordinate system is established, and the coordinate origin is the wearing position of the belt of the slave device, that is, the placement position of the human motion information acquisition module mpu6050.

The fall process can be divided into four stages:

1. In the static and slow walking state, the acceleration in the vertical direction of the human body is 1 g (g represents the gravitational acceleration = 9.8 m/S2);
2. In the fall stage, the human body is in a state of weightlessness, and the value of acceleration becomes smaller;
3. In the impact stage, when the human body collides with the ground, the acceleration value will reach the peak value, and there will be an obvious vibration process in the change trend of acceleration value at this stage.
4. In the static state of complete fall, the human body will be parallel to the ground. At this time, the acceleration value is 1 g. In the process of falling, the acceleration values in three directions will fluctuate greatly.  Figure 9 shows the variation curve of acceleration values in three directions in the process of falling.

As can be seen from Figure 9, the acceleration change law on the three axes is not obvious, which is not conducive to fall analysis. Moreover, when falling in different directions, the acceleration change law of each axis is different. If the acceleration change on each axis is analyzed separately, it is bound to increase the complexity of the algorithm. Therefore, this paper introduces a characteristic quantity SMV (signal magnitude vector) to represent the combined acceleration, which is defined as (14):

(14) $$\begin{array}{c} SMV=\sqrt{a_{x}^{2}+a_{y}^{2}+a_{z}^{2}}. \end{array}$$

SMV is the amplitude of triaxial acceleration vector. Its value has nothing to do with the direction of human movement, but only with the intensity of human movement. Therefore, it can avoid the interference caused by the uncertainty of the falling direction. Select SMV as the acceleration threshold judgment, that is, there is no need to analyze the acceleration change on each axis separately, but it is not rigorous enough to judge the human fall only by the change of combined acceleration, because the system cannot identify whether the current human body is in the state of falling or vigorous exercise, which is prone to wrong judgment. In order to improve the accuracy of the algorithm, the system also introduces the human body inclination for joint judgment, because the human body inclination will change significantly in the process of falling. Generally, when the human body is in the state of complete fall, the inclination angle of the human body is relatively small, between 10 and 25°. Most of the time, the human body is standing, and the inclination of the human body is generally more than 50°. Therefore, by setting the appropriate combined acceleration threshold and human inclination threshold, we can distinguish whether the human body is in the state of falling or vigorous exercise, and the accuracy of fall detection of the system is significantly improved.

RETRACTED

### 4.5. System Test

The process of human fall detection is a complex process. Whether the system can accurately identify and judge the human motion posture, the most critical factor is the accuracy of the fall detection sensor itself and the accuracy of the fall detection algorithm. In the fall simulation experiment of human fall detection module, it is necessary to design the fall simulation experiment of human posture from different directions and angles to detect the accuracy and stability of the fall module. Firstly, carry out statistical experiments, observe and record the change law of human acceleration and angle data through the upper computer, and determine the change law of human acceleration and inclination in the process of falling, so as to lay a foundation for setting a more reasonable threshold in algorithm design. Figures 10 and 11 show the data change trend of acceleration and inclination during one simulated human fall recorded by the upper computer.

Through statistical experiments, we can set a reasonable fall detection algorithm judgment threshold and improve the design of fall detection system. Next, the experiment verifies the accuracy of the system fall detection. The experimenter completes the specified actions related to the fall process according to the instructions. Before each experiment, it must ensure that the Bluetooth communication between the master and slave devices is normal and the master device can send alarm information normally. In order to verify the detection accuracy of this fall detection system, a simple simulation experiment scheme is preliminarily drawn up. The relevant experiments are designed for the two possible results of normal state and fall state: (1) normal state: mainly including normal walking, jogging, and fast sitting; (2) For fall state, the experimenter needs to simulate various possible fall states to verify the detection accuracy of the algorithm. The specific experimental results are shown in Table 2 and Figure 12.

RETRACTED

After testing the main functional modules of the system, it is necessary to debug the whole system, record and observe whether the test results can achieve the expected design objectives. Since serial communication is adopted between many peripheral function modules and Microcontrollers in the hardware design of the system, the host computer can observe the corresponding data flow in cooperation with serial port debugging during the debugging of the whole system. The system test results show that the remote health monitoring system can continuously monitor the heart rate and body temperature all day, and the collected data results are accurate, stable, and reliable. The system can automatically turn on the satellite positioning function when the user's physical sign parameters are abnormal or the user's current fall dangerous situation occurs, and send the current position information and alarm content information through the GSM module, so that the dangerous situation can be found and handled at the first time.

## 5. Conclusion

This paper proposes the detection and application of wearable devices based on the Internet of things in human physical health, and summarizes the related technologies. The module function test and whole machine test of the remote health monitoring system based on wearable devices are carried out. Firstly, the heart rate acquisition module and fall detection module are experimentally verified, and the results are analyzed in detail. Finally, the commissioning test of the whole system is completed to verify the abnormal alarm mechanism of the system. In the research and design of the system, at present, the basic human body sign information data collection and fall detection are completed, and the positioning and alarm information are sent to achieve the expected goal of the subject. In today's world of Internet, the system should expand more cloud services in the future and upload the device detection data to the server for users to view relevant information on the PC or mobile app. In the follow-up research, we should start to improve the accuracy of fall detection algorithm. Continue to explore and study the human posture recognition algorithm and multi-channel data fusion algorithm, and realize the corresponding improvement and innovation on the existing algorithm.

## Figures and Tables

**Figure 1:** Schematic diagram of software development platform.

RETRACTED

**Figure 2:** Schematic diagram of optimal hyperplane of support vector machine.

**Figure 3:** Denoising results of SCDAE model test set.

**Figure 4:** Denoising results of SCDAE model prediction set.

**Figure 5:** Comparison of SNR results after signal denoising.

**Figure 6:** Comparison of r-coefficient results after signal denoising.

**Figure 7:** Software development flow chart.

**Figure 8:** Software design block diagram of wrist strap terminal node based on MSP432.

**Figure 9:** Change of acceleration on three axes during falling.

**Figure 10:** Variation trend of human acceleration.

**Figure 11:** Variation trend of human body inclination.

**Figure 12:** Result of correct rate of fall experiment.

**Table 1:** Denoising results of the SCDAE model.

Record	Test set			Prediction set		
	Baseline drift	Motion artifact	EMG interference	Baseline drift	Motion artifact	EMG interference
SNR	23.3734	20.0069	20.5051	22.1319	18.8539	19.6139
MAE	0.0358	0.0569	0.0549	0.0441	0.0677	0.0544
RMSE	0.0279	0.0419	0.0389	0.0333	0.0468	0.0389
R-square	0.9361	0.8479	0.8821	0.9262	0.8289	0.9121

**Table 2:** Fall test results.

Event	Numberof experiments	Numberof alarms	Accuracy/%
Normal walking	50	1	97
Jogging	50	2	95
Sit down quickly	50	3	93
Fall forward	50	47	95
Fall back	50	46	93
Lateral fall	50	47	95

## Data Availability

No data were used to support this study.
